# Changes of Intestinal Flora and Its Relationship with Nutritional Status for Patients with Cancer Pain

This article has been retracted.

**DOI:** 10.1155/2022/5188202

**Published:** 2022-08-17

**Authors:** Ping Zhang, Na Zhu, Ping Wang, Feifei Zhuang, Daihong Ding, Dongmei Zhou

**Affiliations:** Department of Oncology, Yantai Mountain Hospital, Yantai City, Shandong Province, China

## Abstract

**Objective:**

To study the changes in the intestinal flora and its relationship with nutritional status for patients with cancer pain.

**Methods:**

A prospective research method was adopted. One hundred twenty cancer patients with cancer pain were selected as the research objects, who were treated in our hospital from June 2019 to June 2020, and 120 cancer patients without cancer pain were selected as the control group, who were treated in the same period. The differences of the intestinal flora and nutritional status of patients with different severity between the observation group and the control group were compared to analyze the changes of intestinal flora in patients with cancer pain and its correlation with nutritional status.

**Results:**

Hemoglobin (HB) (*t* = 17.141, *p* ≤ 0.001), albumin (ALB) (*t* = 27.654, *p* ≤ 0.001), prealbumin (PAB) (*t* = 96.192, *p* ≤ 0.001), and total protein (TP) (*t* = 18.781, *p* ≤ 0.001) in the observation group were significantly lower than those in the control group. There were statistically significant differences in HB (*f* = 13.569, *p* ≤ 0.001), ALB (*f* = 22.229, *p* ≤ 0.001), PAB (*f* = 19.521, *p* ≤ 0.001), and TP (*f* = 21.451, *p* ≤ 0.001) among patients with cancer pain of different severity. Through these two comparisons, their nutritional indicators showed a significant downward trend with the increase in the severity for cancer pain patients; the levels of Lactobacillus (*t* = 2.124, *p* = 0.035), Bifidobacterium (*t* = 4.823, *p* ≤ 0.001), Enterococcus (*t* = 3.578, *p* ≤ 0.001), and Eubacterium (*t* = 2.394, *p* = 0.017) in the observation group were significantly lower than those in the control group. There were statistically significant differences in the levels of Lactobacillus (*f* = 20.643, *p* ≤ 0.001), Bifidobacterium (*f* = 19.129, *p* ≤ 0.001), Enterococcus (*f* = 17.408, *p* ≤ 0.001), and Eubacterium (*f* = 22.343, *p* ≤ 0.001) among patients with cancer pain of different severity. After pairwise comparison, their beneficial intestinal bacteria were significantly lower than those in the control group with the increase in pain in cancer pain patients. Nitric oxide (NO) (*t* = 8.418, *p* ≤ 0.001), galectin-3 (*t* = 14.043, *p* ≤ 0.001), occludin (OCLN) (*t* = 47.308, *p* ≤ 0.001), galectin-1 (*t* = 15.298, *p* ≤ 0.001), zonula occludens protein 1 (ZO-1) (*t* = 23.093, *p* ≤ 0.001), and cingulin (*t* = 340.198, *p* ≤ 0.001) in the observation group were significantly lower than those in the control group. There were statistically significant differences in NO, galectin-3, OCLN, galectin-1, ZO-1, and cingulin for patients with cancer pain of different severity. By comparison, the NO, galectin-3, OCLN, galectin-1, ZO-1, and cingulin of the patients showed a significant downward trend with the aggravation of cancer pain symptoms. Through correlation analysis, the nutritional indicators of patients were positively correlated with intestinal microorganisms and intestinal barrier function.

**Conclusion:**

There was a significant correlation between the changes in intestinal flora and nutritional status for patients with cancer pain, which could be used as an important basis for improving the treatment of cancer pain.

## 1. Introduction

According to the survey of the World Health Organization [1], the global incidence rate of cancer patients showed a significant upward trend. With the development of diagnosis and treatment, tumor disease has become a controllable and even curable chronic disease. The course of this disease was long [2]. In treating patients, the method had become the focus of common clinical attention, which could significantly improve patients' quality of life through active and effective early intervention and treatment measures [3]. According to the national comprehensive cancer network of the United States [4], there was cancer pain for 25% of patients with new malignant tumors, more than 33% of patients with treated malignant tumors, and 75% of patients with malignant tumors. In the progress of advanced malignant tumor diseases, the appetite decreased significantly with the invasion of malignant tumors to the digestive tract, and the absorption capacity of nutrients decreased significantly [5]. At the same time, painful stimulation increases the excitability of the sympathetic nervous system, reduces the tone of the smooth muscles of the gastrointestinal tract, increases the tone of the sphincter, and significantly enhances the feeling of fullness, which will affect the patient's appetite and eventually lead to malnutrition [6].

Meanwhile, the stress response caused by pain would also cause the secretion of catechol, adrenergic hormone, glucagon, and cortisol to decrease, further affecting the metabolism of intestinal glycogen, protein, and lipid. The intestinal flora of the body presented a corresponding disorder with the influence of metabolic disorder, thus affecting the nutritional status of patients [7]. This study mainly analyzed the changes in the intestinal flora and its relationship with the nutritional status of patients with cancer pain to guide clinical treatment.

## 2. Data and Methods for This Research

### 2.1. General Information

A prospective research method was adopted for this study. One hundred twenty cancer pain patients treated in our hospital from June 2019 to June 2020 were selected as the research objects, including 57 male patients and 63 female patients aged 45-59 years, with an average age of 55.69 ± 2.47 years, an average body mass index of 24.55 ± 5.41 kg/m^2^, and an average length of education of 14.65 ± 2.51 years. There were 25 cases of gastric cancer, 41 cases of lung cancer, 34 cases of liver cancer, and 20 cases of colorectal cancer. According to the numerical scoring system (NRS), 1-3 points were mild pain, 4-6 points were moderate pain, and 7-10 points were severe pain; there were 35 cases with mild pain, 40 cases with moderate pain, and 45 cases with severe pain. In addition, 120 cancer patients without cancer pain treated in the same period were selected as the control group. There was no significant difference between the general data of the two groups (*p* > 0.05), as shown in Table 1. All patients signed the informed consent form, which the ethics committee approved. All patients in this study have completed this study, and no patients have dropped out of the study halfway.

The inclusion criteria were as follows: (1) all patients met the diagnostic criteria for cancer pain [8]; (2) all patients were diagnosed by imaging; (3) the duration of cancer pain in all patients was more than 1 week; and (4) patients are expected to live longer than 3 months. Also, the exclusion criteria were as follows: (1) AIDS patients, (2) trauma patients, (3) patients with cognitive impairment, (4) patients with incomplete clinical information, and (5) patients with pain caused by other diseases.

### 2.2. The Method for This Research

The analysis of nutritional indicators was performed: 5 ml of fasting blood was collected after all patients were enrolled in the group. The levels of hemoglobin (HB), albumin (ALB), prealbumin (PAB), and total protein (TP) were detected with an automatic biochemical instrument.

Then, intestinal microbiota was analyzed: all patients were tested for feces after enrollment. The NEB DNA assay was used to compare the number of Bifidobacteria, Enterococcus, Lactobacillus, and Eubacterium.

At last, the detection of intestinal barrier function was carried out: the colon epithelial tissue of the patient was taken as the research object by colonoscopy, and the abrasive treatment solution of the above samples was lysed with RIRP lysate. At the same time, after centrifugation at 1000 r/min for 10 min, the upper liquid was taken, and the above liquid was subjected to nitric oxide (NO). Meanwhile, galectin-3, occludin (OCLN), galectin-1, zonula occludens protein 1 (ZO-1), and cingulin were analyzed.

### 2.3. Observation Indicators

There was a comparison of nutritional indexes between the observation group and the control group. The levels of Hb, ALB, PAB, and TP in the observation group and the control group were compared.

There was a comparison of nutritional indicators for patients with cancer pain of different severity. The levels of Hb, ALB, PAB, and TP in patients with mild, moderate, and severe cancer pain were compared.

There was a comparison of intestinal microorganisms between the observation and control groups. The numbers of Bifidobacterium, Enterococcus, Lactobacillus, and Eubacterium in the observation group and the control group were compared.

There was a comparison of intestinal microorganisms in patients with cancer pain of different severity. The numbers of Bifidobacterium, Enterococcus, Lactobacillus, and Eubacterium in patients with mild, moderate, and severe cancer pain were compared.

There was a comparison of intestinal barrier function between the observation and control groups. The levels of NO, galectin-3, OCLN, galectin-1, ZO-1, and cingulin in the observation and control groups were compared.

There was a comparison of intestinal barrier function in patients with cancer pain of different severity. The levels of NO, galectin-3, OCLN, galectin-1, ZO-1, and cingulin in patients with mild, moderate, and severe cancer pain were compared.

There was a correlation analysis. Linear correlation was used to analyze the correlation between intestinal flora, intestinal barrier, and nutritional status.

### 2.4. Statistical Method

The data in this paper were collected and analyzed by SPSS 20.0 software. All the research data were positive distribution, where the measurement data were expressed as $\bar{x}\pm s$, and the counting data were expressed as *n* (%). The difference was statistically significant when *p* < 0.05.

## 3. Results of the Research

### 3.1. Comparison of Nutritional Indexes between the Observation Group and Control Group

HB (*t* = 17.141, *p* ≤ 0.001), ALB (*t* = 27.654, *p* ≤ 0.001), PAB (*t* = 96.192, *p* ≤ 0.001), and TP (*t* = 18.781, *p* ≤ 0.001) in the observation group were significantly lower than those in the control group, as shown in Table 2.

### 3.2. Comparison of Nutritional Indicators in Patients with Cancer Pain of Different Severity

There were statistically significant differences in HB (*f* = 13.569, *p* ≤ 0.001), ALB (*f* = 22.229, *p* ≤ 0.001), PAB (*f* = 19.521, *p* ≤ 0.001), and TP (*f* = 21.451, *p* ≤ 0.001) among patients with cancer pain of different severity. Through pairwise comparison, the nutritional indicators showed a significant downward trend with the increase in cancer pain severity, as shown in Table 3.

### 3.3. Comparison of Intestinal Microorganisms between the Observation Group and the Control Group

Lactobacillus (*t* = 2.124, *p* = 0.035), Bifidobacterium (*t* = 4.823, *p* ≤ 0.001), Enterococcus (*t* = 3.578, *p* ≤ 0.001), and Eubacterium (*t* = 2.394, *p* = 0.017) in the observation group were significantly lower than those in the control group, as shown in Table 4.

### 3.4. Comparison of Intestinal Microorganisms in Patients with Cancer Pain of Different Severity

There were statistically significant differences in Lactobacillus (*f* = 20.643, *p* ≤ 0.001), Bifidobacterium (*f* = 19.129, *p* ≤ 0.001), Enterococcus (*f* = 17.408, *p* ≤ 0.001), and Eubacterium (*f* = 22.343, *p* ≤ 0.001) among patients with cancer pain of different severity. After pairwise comparison, their beneficial intestinal bacteria were significantly lower than those in the control group with an increase in pain in cancer patients, as shown in Table 5.

### 3.5. Comparison of Intestinal Barrier Function between the Observation Group and Control Group

NO (*t* = 8.418, *p* ≤ 0.001), galectin-3 (*t* = 14.043, *p* ≤ 0.001), OCLN (*t* = 47.308, *p* ≤ 0.001), galectin-1 (*t* = 15.298, *p* ≤ 0.001), ZO-1 (*t* = 23.093, *p* ≤ 0.001), and cingulin (*t* = 340.198, *p* ≤ 0.001) in the observation group were significantly lower than those in the control group, as shown in Table 6.

### 3.6. Comparison of Intestinal Barrier Function in Patients with Cancer Pain of Different Severity

There were statistically significant differences in NO, galectin-3, OCLN, galectin-1, ZO-1, and cingulin in patients with cancer pain of different severity. By comparison, NO, galectin-3, OCLN, galectin-1, ZO-1, and cingulin showed a significant downward trend with the aggravation of cancer pain symptoms, as shown in Table 7.

### 3.7. Correlation Analysis

Through correlation analysis, the nutritional indicators of patients were positively correlated with intestinal microorganisms and intestinal barrier function, as shown in Table 8.

## 4. Conclusion

Malnutrition was one of the common clinical complications. Some research reports showed that [9], in treating tumor diseases, if patients had nutritional risk or malnutrition, it would seriously affect the prognosis of patients. In the progress of tumor diseases, patients' pain mainly included their actual feelings about the disease and potential tissue damage [10]. In the progress of the tumor, the body also faces the interference of negative emotions in addition to the body's pain. Due to excessive worry, sadness, and fear of the disease [11, 12], the possibility of psychological disorders was significantly increased. Previous studies had pointed out that the detection rate of psychological pain could reach more than 35% in the study of patients with tumor diseases [13–15]. Psychological pain was often ignored in clinical practice, but in the study of patients, psychological pain often caused the pain of clinical organisms. With the significant improvement of inflammatory reaction and oxidative stress reaction at the focus [16], gastrointestinal spasms and abnormal excitation of sympathetic nerves in patients further led to the occurrence of malnutrition in the body, forming a vicious circle, which had a negative impact on the prognosis of patients [17].

In this study, through the analysis of the nutritional indicators and intestinal microbial conditions of the patients between the observation group and the control group, the nutritional indicators and intestinal microbial conditions of the patients in the observation group were significantly lower than those in the control group. At the same time, the nutritional indicators and intestinal microbial conditions of the patients showed a significant downward trend with a significant increase in cancer pain. During the invasion of tumor cells into surrounding tissues, it was bound to cause a significant increase in the level of inflammatory response and oxidative stress response in the above regional tissues [18, 19]. In the digestive tract, the patient's mucosa was correspondingly damaged, and the ability to absorb nutrients was significantly reduced [20]. The body's vitamin D level was significantly deficient, and the risk of diffuse muscle pain in the waist, pelvis, and lower limbs was significantly increased [21]. It had been confirmed in foreign studies [22–24] that the level of 25 hydroxyvitamin D showed a significant correlation with the dosage of opioids in tumor patients. The low serum magnesium level was also an important reason for the decrease in opioid sensitivity [25]. In animal experiments [26], aspartate receptors had a significant correlation with the tolerance of opioids. Magnesium ion was an important antagonist of this receptor. With the significant reduction of digestion capacity, the absorption capacity of magnesium ion level decreased significantly [27, 28]. Therefore, in the study of cancer pain patients, it could further cause a significant increase in their pain index through the impact on the nutritional indicators of the digestive tract. The osmotic pressure of local tissues changes significantly with the spasm of the body's intestinal muscles in the analysis of the patient's intestinal flora and intestinal barrier function [29]. At the same time, the change of intestinal flora was obvious with the influence of negative emotions, which had a negative impact on the absorption of nutrients [30]. Nitric oxide reflected the osmotic pressure of the intestinal mucosa in the body to some extent, while galectin-1 and galectin-3 reflected the levels of vascular endothelial growth factor and basic fibroblast growth factor [31]. OCLN was an important indicator of the intestinal inflammatory response [32]; cingulin and ZO-1 were important indicators of the gap between intestinal cells [33], through the influence on the tissue arrangement of intestinal mucosal cells, further affecting the intestinal osmotic pressure [34]. Through the correlation analysis, the intestinal flora and intestinal barrier of patients were significantly correlated with nutritional indicators, suggesting that in the treatment of cancer pain patients, the quality of life of patients could be further improved through the adjustment of intestinal flora or nutritional intervention [35].

There are also some shortcomings in this study. The patients in this study are all from the same hospital, which is not representative of the patient's overall situation and will lead to some bias in the results. This study only found that changes in the gut microbiota of cancer pain patients are related to nutritional status, but which type of flora plays an important role, how does it work, and whether it is metabolites or other pathways have not been studied in depth. In addition, this study only studies several microbiotas. With the development of the microbiome, sequencing into an effective method can detect the various flora changes in the patient's body; through sequencing, there will be more accurate detailed results.

In conclusion, there was a significant correlation between the changes in the intestinal flora and nutritional status for patients with cancer pain, which could be used as an important basis for improving the treatment of cancer pain.

## Figures and Tables

**Table 1:** Comparison of baseline data between the two groups.

Group	Gender (male/female)	Age (years)	Body mass index (kg/m^2^)	Years of education (years)	Lesion location (stomach/lung/liver/colorectal)
Observation group (*n* = 120)	57/63	55.69 ± 2.47	24.55 ± 5.41	14.65 ± 2.51	25/41/34/20
Control group (*n* = 120)	53/67	55.81 ± 3.52	24.94 ± 5.33	14.59 ± 1.49	25/45/30/20
*χ* ^2^/*t*	0.269	0.306	0.563	0.225	0.436
*p*	0.604	0.760	0.574	0.822	0.933

**Table 2:** Comparison of nutritional indexes between the observation group and control group.

Group	HB (g/L)	ALB (g/L)	PAB (mg/L)	TP (g/L)
Control group (*n* = 120)	119.63 ± 3.48	52.02 ± 2.72	314.81 ± 3.87	67.77 ± 2.45
Observation group (*n* = 120)	112.42 ± 3.02	41.36 ± 3.23	272.08 ± 2.95	61.57 ± 2.66
*t*	17.141	27.654	96.192	18.781
*p*	<0.001	<0.001	<0.001	<0.001

**Table 3:** Comparison of nutritional indicators in patients with cancer pain of different severity.

Group	HB (g/L)	ALB (g/L)	PAB (mg/L)	TP (g/L)
Mild group (*n* = 35)	114.89 ± 2.96	45.46 ± 2.52	280.26 ± 3.66	65.54 ± 3.33
Moderate group (*n* = 40)	112.51 ± 3.44	41.17 ± 2.99	272.17 ± 3.77	61.48 ± 2.98
Severe group (*n* = 45)	110.28 ± 3.63	37.63 ± 2.97	265.75 ± 3.83	57.55 ± 2.86
*f*	13.569	22.229	19.521	21.451
*p*	<0.001	<0.001	<0.001	<0.001
LSD-t (mild vs. moderate)	16.384	20.951	15.164	14.134
*p*	<0.001	<0.001	<0.001	<0.001
LSD-t (mild vs. severe)	16.331	14.148	14.728	19.499
*p*	<0.001	<0.001	<0.001	<0.001
LSD-t (severe vs. moderate)	14.539	22.327	21.178	17.964
*p*	<0.001	<0.001	<0.001	<0.001

**Table 4:** Comparison of intestinal microorganisms between the observation group and control group.

Group	Lactobacillus (CFU)	Bifidobacterium (CFU)	Enterococcus (CFU)	Eubacterium (CFU)
Control group (*n* = 120)	8.81 ± 2.45	10.54 ± 2.74	8.98 ± 3.26	8.93 ± 2.72
Observation group (*n* = 120)	8.01 ± 3.32	8.91 ± 2.49	7.64 ± 2.49	8.16 ± 2.24
*t*	2.124	4.823	3.578	2.394
*p*	0.035	<0.001	<0.001	0.017

**Table 5:** Comparison of intestinal microorganisms in patients with cancer pain of different severity.

Group	Lactobacillus (CFU)	Bifidobacterium (CFU)	Enterococcus (CFU)	Eubacterium (CFU)
Mild group (*n* = 35)	8.22 ± 0.61	8.99 ± 0.63	8.49 ± 0.99	8.83 ± 0.94
Moderate group (*n* = 40)	8.01 ± 0.32	8.85 ± 0.95	7.65 ± 0.86	8.22 ± 0.64
Severe group (*n* = 45)	7.88 ± 0.52	8.62 ± 0.75	7.48 ± 0.91	7.95 ± 0.33
*f*	20.643	19.129	17.408	22.345
*p*	<0.001	<0.001	<0.001	<0.001
LSD-t (mild vs. moderate)	13.699	18.662	22.346	12.772
*p*	<0.001	<0.001	<0.001	<0.001
LSD-t (mild vs. severe)	15.737	15.096	14.398	16.701
*p*	<0.001	<0.001	<0.001	<0.001
LSD-t (severe vs. moderate)	18.763	19.025	18.401	13.002
*p*	<0.001	<0.001	<0.001	<0.001

**Table 6:** Comparison of intestinal barrier function between the observation group and control group.

Group	NO (U/L)	Galectin-3 (ng/mL)	OCLN (pg/mL)	Galectin-1 (ng/mL)	ZO-1 (ng/mL)	Cingulin (pg/mL)
Control group (*n* = 120)	15.92 ± 3.11	7.72 ± 1.82	426.26 ± 3.55	11.3 ± 2.53	4.92 ± 1.11	363.7 ± 2.18
Observation group (*n* = 120)	12.27 ± 3.59	5.02 ± 1.06	406.92 ± 2.73	7.48 ± 1.04	2.27 ± 0.59	247.02 ± 3.06
*t*	8.418	14.043	47.308	15.298	23.093	340.198
*p*	<0.001	<0.001	<0.001	<0.001	<0.001	<0.001

**Table 7:** Comparison of intestinal barrier function in patients with cancer pain of different severity.

Group	NO (U/L)	Galectin-3 (ng/mL)	OCLN (pg/mL)	Galectin-1 (ng/mL)	ZO-1 (ng/mL)	Cingulin (pg/mL)
Mild group (*n* = 35)	13.18 ± 2.88	5.25 ± 2.72	411.94 ± 3.98	8.45 ± 1.95	2.43 ± 0.15	255.93 ± 3.9
Moderate group (*n* = 40)	12.13 ± 2.96	6.71 ± 3.71	406.13 ± 3.56	7.42 ± 1.48	2.21 ± 0.37	247.23 ± 2.93
Severe group (*n* = 45)	11.79 ± 1.92	7.22 ± 1.29	400.11 ± 2.57	6.68 ± 1.07	2.02 ± 0.63	235.64 ± 2.52
*f*	13.414	20.385	22.175	14.629	12.958	15.192
*p*	<0.001	<0.001	<0.001	<0.001	<0.001	<0.001
LSD-t (mild vs. moderate)	14.949	18.554	18.717	15.135	14.766	14.881
*p*	<0.001	<0.001	<0.001	<0.001	<0.001	<0.001
LSD-t (mild vs. severe)	16.171	17.098	12.866	14.043	20.774	20.181
*p*	<0.001	<0.001	<0.001	<0.001	<0.001	<0.001
LSD-t (severe vs moderate)	13.651	22.081	18.302	14.392	19.802	18.232
*p*	<0.001	<0.001	<0.001	<0.001	<0.001	<0.001

**Table 8:** Correlation analysis.

Index		NO	Galectin-3	OCLN	Galectin-1	ZO-1	Cingulin	Lactobacillus	Bifidobacterium	Enterococcus	Eubacterium
HB	*r*	0.666	0.591	0.723	0.506	0.681	0.633	0.709	0.448	0.688	0.666
	*p*	<0.001	<0.001	<0.001	<0.001	<0.001	<0.001	<0.001	<0.001	<0.001	<0.001
ALB	*r*	0.648	0.64	0.883	0.344	0.842	0.761	0.43	0.775	0.812	0.648
	*p*	<0.001	<0.001	<0.001	<0.001	<0.001	<0.001	<0.001	<0.001	<0.001	<0.001
PAB	*r*	0.65	0.726	0.653	0.722	0.555	0.426	0.517	0.736	0.784	0.65
	*p*	<0.001	<0.001	<0.001	<0.001	<0.001	<0.001	<0.001	<0.001	<0.001	<0.001
TP	*r*	0.559	0.783	0.395	0.722	0.526	0.402	0.828	0.443	0.56	0.559
	*p*	<0.001	<0.001	<0.001	<0.001	<0.001	<0.001	<0.001	<0.001	<0.001	<0.001

## Data Availability

The datasets used and analyzed during the current study are available from the corresponding author upon reasonable request.
